The article "Hemodynamic and Geometric Risk Factors for In-Stent Restenosis in Patients with Intracranial Atherosclerotic Stenosis" was retracted in 2024. Reasons: signs of a paper mill; suspected computer-generated content; unreliable results or conclusions; concerns about the data.

# Hemodynamic and Geometric Risk Factors for In-Stent Restenosis in Patients with Intracranial Atherosclerotic Stenosis

**DOI:** 10.1155/2022/6951302

**Published:** 2022-07-27

**Authors:** Xiaowen Song, Hancheng Qiu, Shuo Wang, Yong Cao, Jizong Zhao

**Affiliations:** ^1^Department of Neurosurgery, Beijing Tiantan Hospital, Capital Medical University, Beijing, China; ^2^China National Clinical Research Center for Neurological Diseases, Beijing, China; ^3^Center of Stroke, Beijing Institute for Brain Disorders, Beijing, China; ^4^Beijing Key Laboratory of Translational Medicine for Cerebrovascular Disease, Beijing, China

## Abstract

**Methods:**

Severe ICAS patients managed with percutaneous transluminal angioplasty and stenting (PTAS) were included in the retrospective cohort study and were divided into two groups according to whether ISR occurred at follow-up (ISR group and no-ISR group). Computational fluid dynamics models were built based on digital subtraction angiography before and after PTAS to simulate blood flow and quantify hemodynamic parameters. The associations between vessel geometry, hemodynamics, and ISR in ICAS patients were investigated.

**Results:**

Among 39 patients, ISR occurred in seven patients (17.95%) after a mean follow-up period of 6.69 ± 3.24 months. Stenting decreased vessel angulation (51.11° [40.07°–67.27°] vs. 15.97° [0.00°–36.16°], *P* = 0.000) and vessel tortuosity (0.09 [0.06–0.13] vs. 0.01 [0.00–0.03], *P* = 0.000). Meanwhile, the translational pressure ratio (PR) dramatically increased (0.07 [0.00–0.31] vs. 0.62 [0.41–0.82], *P* = 0.000) with the wall shear stress ratio decreased (13.93 [8.37–40.30] vs. 2.90 [1.69–4.48], *P* = 0.000). In the multivariate analysis, smaller Δ tortuosity (*P* = 0.038) was independently associated with the occurrence of ISR, and smaller post-PTAS translesional PR was also a predictive factor of marginal significance (*P* = 0.059).

**Conclusion:**

PTAS decreased vessel angulation, vessel tortuosity, and translesional wall shear stress ratio while it increased translesional pressure ratio (PR) dramatically in ICAS patients. Smaller Δ tortuosity was found to be a risk factor for ISR, and smaller post-PTAS translesional PR was also a predictive factor of marginal significance, indicating that both geometric and hemodynamic parameters played important roles in the occurrence of ISR after PTAS.

## 1. Introduction

Hemodynamic factors had a profound influence on vascular physiology and homeostasis, thus playing important roles in the development and progression of various vascular diseases such as atherosclerosis or stenosis [1]. Vessel geometry had been proven to affect the blood flow pattern through the artery, regulating the function of arterial endothelium and attributing to atherosclerotic stenosis [2].

Intracranial atherosclerotic stenosis (ICAS) was a major ischemic stroke subtype of high recurrence, causing approximately 5% to 10% of strokes in White people, 15% to 29% of transient ischemic attacks (TIAs) or strokes in Black people, and up to 30% to 50% of strokes in Asian people [3]. For patients with high-grade ICAS, despite optimal medical treatment, the risk of recurrent stroke that might result from embolic events and hemodynamic insufficiency was as high as 12.6% in the SAMMPRIS (Stenting and Aggressive Medical Management for Preventing Recurrent Stroke in Intracranial Stenosis) trial [4] and 23% in the WASID (Warfarin-Aspirin Symptomatic Intracranial Disease) trial during the first year [5]. For Chinese population, the rate of recurrent stroke within 3 months could be 11.3% for ICAS patients with aggressive medical treatment [6].

Percutaneous transluminal angioplasty and stenting (PTAS) had emerged as a possible treatment option. With a 2.6% periprocedural stroke and death rate, the WEAVE (Wingspan StEnt System Post MArket SurVEillance) trial revealed the excellent safety and efficiency of this treatment [7]. Stenting could not only normalize the lumen diameter but also change the geometry of target vessels, resulting in underlying hemodynamic alterations. However, the hemodynamic influences of PTAS in small-caliber intracranial vessels had not been well demonstrated [8–10].

In the long term, clinicians should pay attention to challenges such as restenosis or delayed stent thrombosis after PTAS. With a 6.81% to 31.18% occurrence rate [11–19], the in-stent restenosis (ISR) in ICAS might be affected by features of the lesion and characteristics of the stent, which was controversial and not definite [11, 15, 16, 20]. In carotid and coronary arteries, local hemodynamic changes caused by geometric variations had been suggested to govern the risk and mechanism of ISR [21–24]. However, the hemodynamic and geometric features prone to adverse events, especially ISR in ICAS, had never been studied before.

This current study sought to evaluate the geometrical and hemodynamic changes caused by PTAS using computational fluid dynamic (CFD) analysis of patient-specific digital subtraction angiography (DSA) data, delineate associations between hemodynamics and vessel geometry, and identify hemodynamic and geometric factors implicated in the initiation and progression of ISR.

## 2. Materials and Methods

### 2.1. Patient Selection

This was a retrospective cohort study. We retrospectively screened eligible patients admitted to Beijing Tiantan Hospital from January 2020 to June 2021. Thirty-nine adult patients with severe ICAS (70%–99%) treated with PTAS were identified according to the following criteria: (1) history of ischemic stroke or TIA attributed to 70% to 99% atherosclerotic stenosis of a major intracranial artery (intracranial portion of the internal carotid artery (ICA), M1 middle cerebral artery (MCA-M1), V4 vertebral artery (VA-V4), or basilar artery (BA)), as revealed by DSA; (2) computed tomography perfusion imaging showing apparent hypoperfusion in the corresponding territory of the target intracranial artery; and (3) receiving PTAS for the severe ICAS. We excluded patients with the following conditions: (1) the index ischemic stroke or TIA was attributed to nonatherosclerotic intracranial arterial stenosis such as moyamoya disease, vasculitis or dissection, restenosis within a stented artery, or tandem stenosis of extracranial and intracranial arteries; (2) there was any potential cardioembolic source; and (3) there was known intracranial tumor, arteriovenous malformation, or aneurysm.

Patients' demographics, history of common cardiovascular risk factors, onset symptoms, lesion locations, and stroke severity by the National Institutes of Health Stroke Scale were obtained from electronic medical database. In each case, geometric metrics were assessed on three-dimensional- (3D-) DSA images, and a CFD model was built based on DSA images before and after PTAS to quantify the hemodynamic features.

This retrospective study was in accordance with the 1964 Helsinki Declaration and its later amendments or comparable ethical standards, and the research flow chart is shown in Figure 1. Informed consent was waived by the ethics committee of Beijing Tiantan Hospital because of the retrospective nature of the study (KY2016-034-02).

### 2.2. Treatment and Follow-Up

All patients had been pretreated with dual antiplatelet therapy (aspirin 300 mg and clopidogrel 75 mg daily) started at least 5 days before stenting. The PTAS procedures were successfully fulfilled using self-expanding stents by highly experienced neurosurgeons. After stent deployment, patients were maintained on dual antiplatelet therapy for at least 3 months, which was replaced by antiplatelet monotherapy (aspirin or clopidogrel) afterward.

According to the standard follow-up regimen after PTAS at our center, initial follow-up angiography would be performed at 3 to 12 months following the stent deployment procedure in all included patients. Further follow-up or treatment would be performed as dictated by clinical symptoms and findings on the initial angiogram. The follow-up DSA images were collected from the radiological database for ISR evaluation. If the luminal narrowing in the affected vessel was greater than 50%, it would be considered restenosis.

### 2.3. Assessment of Geometric Features

Patient-specific models were reconstructed from pre- and post-PTAS DSA source images for further quantitative analysis. Multiplanar reconstructions were oriented at the working angles for stenting to enable the measurement. Centerlines of the interested vessels were generated in 3-Matic from the catheter 3D rotational angiography. The vessel angulation was referred to as the angle between the local vessel centerlines of the proximal and distal vessels to the local stenosis (Figure 2). Angles were measured in the direction of the flow. As shown in Figure 3, vessel tortuosity was defined as *T*/*D* − 1, where *T* was the length of the centerline between two points proximal and distal to the local stenosis and *D* was the straight-line distance between these 2 points [25, 26]. Geometric parameters were measured before and after stenting and at subsequent angiographic follow-up. The differences of vessel tortuosity and angulation between pre- and post-PTAS defined as Δ tortuosity and Δ angulation were calculated, respectively.

### 2.4. CFD Modeling and Quantification of Hemodynamic Features of ICAS

CFD analysis was performed using the patients' 3D-DSA data before and after stenting for comparison of hemodynamic alteration caused by PTAS. 3D geometry of the arteries of interest was reconstructed from DSA source images with Mimics and Magics, covering the ICA; MCA-M1, M2; and ACA-A1, A2 segments for cases with ICA or MCA-M1 lesion and VA-V4, BA, PCA-P1 segments and SCA for cases with a VA-V4 or BA lesion. A mesh was then created on the vessel surface in ANSYS ICEM CFD, with the maximal element sizes of 0.1 for the inlet(s) and outlets and 0.2 for other parts of the mesh, containing at least 1 million elements in total for each case. The procedure of CFD modeling was shown in Figure 4. Blood flow simulation was performed on this mesh using ANSYS CFX software. The following settings and assumptions were applied in simulation of the blood flow: (1) rigid, noncompliant walls with no-slip boundary conditions were assumed; (2) the outlet pressure was set to be 0 Pa, as we primarily focused on the relative translesional pressure change across the ICAS lesion; (3) the individualized mean flow velocity at the inlet was obtained from each patient's transcranial Doppler; (4) blood flow simulation was conducted in ANSYS CFX by solving the Navier-Stokes equations; convergence was achieved when the root mean square residual value reached below 10^−4^; and (5) blood was an incompressible Newtonian fluid with a constant viscosity of 0.0035 kg/(m∗s) and a density of 1060 kg/m^3^.

We quantified the relative changes of pressure and wall shear strain (WSS) across each ICAS lesion, by obtaining translesional pressure ratio (PR) and WSS ratio (WSSR) on the CFD models in ANSYS CFD-post. In the pre-PTAS model, translesional PR was calculated as pressure_poststenotic_/pressure_prestenotic_, and pressure_poststenotic_ and pressure_prestenotic_ were measured at the first normal diameter distal to the ICAS lesion and at the proximal normal vessel segment, respectively. Translesional WSSR was calculated as WSS_stenotic−apex_/WSS_prestenotic_;, and WSS_stenotic-apex_ was measured at the most severely narrowed cross-section of the diseased intracranial artery referred to as the stenotic throat, and WSS_prestenotic_ was measured at the proximal normal vessel segment. In the post-PTAS model, these hemodynamic indices were measured at the correspondingly the same locations as in the pre-PTAS model. The difference between pre- and post-PTAS hemodynamic features was calculated.

### 2.5. Statistical Analysis

Continuous variables and ordinal variables (National Institutes of Health Stroke Scale) were expressed as median and interquartile range, and frequency and categorical variables were expressed as the frequency and percentage. We compared the geometric and hemodynamic metrics between pre- and post-PTAS by Wilcoxon rank sum test. The Mann–Whitney *U* test was used for univariable comparisons of continuous variables and *χ*^2^ tests or Fisher exact test for categorical variables between patients with ISR and no-ISR during follow-up period. Nonparametric tests were adopted while needed. Multivariate logistic regression model was established to predict ISR, adjusting for other factors with *P* < 0.1 in univariate logistic regression. In addition, we analyzed the associations between geometric and hemodynamic features by using Spearman correlation coefficients. We considered *P* < 0.05 as statistically significant. We conducted all statistical analyses in IBM SPSS Statistics version 22.0 (IBM Corp, Armonk, New York).

## 3. Results

Among 52 potentially eligible patients with severe ICAS confirmed in DSA who were scheduled a second follow-up DSA at 6 months, we excluded 12 cases with poor DSA image quality or complex vessel geometry that did not allow CFD model construction and one case for failure in solving the Navier-Stokes equations in simulation of blood flow. Therefore, 39 patients were included in the current study (mean age, 57.51 years; 22 males; Table 1). Twenty-two patients (56%) had the ICAS lesion in the anterior circulation (20 in MCA-M1, 2 in intracranial ICA). No difference was found between the baseline characteristics of the ISR and no-ISR group.

As shown in Tables 2–3, at the affected arteries, prominent hemodynamic changes were brought about by PTAS (Figure 5). Translesional PR (0.07 [0.00–0.31] vs. 0.62 [0.41–0.82], *P* = 0.000) increased, whereas WSSR (13.93 [8.37–40.30] vs. 2.90 [1.69–4.48], *P* = 0.000) decreased significantly after PTAS. Besides minimizing the luminal narrowness, stenting straightened the target vessel, significantly decreasing vessel tortuosity (0.01 [0.00–0.03] vs. 0.09 [0.06–0.13], *P* = 0.000) and vessel angulation (15.97° [0.00°–36.16°] vs. 51.11° [40.07°–67.27°], *P* = 0.000).

All patients underwent angiographic follow-up from 3 to 24 months (mean, 6.41 months). After PTAS, the deployed stent exerted a continuous outwardly directed radial force resulting in persistent vascular remodeling. At the angiographic follow-up, a significant difference existed in vessel tortuosity (0.01 [0.00–0.03] vs. 0.09 [0.06–0.13], *P* = 0.000) and angulation (21.46° [0.00°–31.34°] vs. 51.11° [40.07°–67.27°], *P* = 0.000) compared with those measured before PTAS (Figure 6). Nevertheless, when compared with the vessel geometry after PTAS, no significant differences were found (0.01 [0.00–0.03] vs. 0.01 [0.00–0.03], *P* = 0.575; 21.46° [0.00°–31.34°] vs. 15.97° [0.00°–36.16°], *P* = 0.112) (Table 3).

Seven patients (17.95%) were diagnosed with ISR during follow-up. Compared with those without ISR, ICAS lesions with ISR had significantly larger vessel tortuosity (0.06 [0.02–0.10] vs. 0.05 [0.00–0.01], *P* = 0.001) and lower PR (0.36 [0.05–0.62] vs. 0.67 [0.50–0.89], *P* = 0.024) after PTAS. In addition, ISR lesions had smaller Δ tortuosity (0.05 [0.02–0.06] vs. 0.08 [0.06–0.12], *P* = 0.006) and smaller Δ angulation (14.08° [6.00°–29.24°] vs. 33.53° [22.85°–44.05°], *P* = 0.016) (Table 4).

As shown in Table 5, there was a strong linear correlation between translesional PR and WSSR (*r*_s_ = −0.672, *P* = 0.000; *r*_s_ = −0.566, *P* = 0.000) both before and after PTAS (Figure 7). Besides, after PTAS, vessel tortuosity was negatively linearly correlated with PR (*r*_s_ = −0.673, *P* = 0.000) and positively with WSSR (*r*_s_ = 0.547, *P* = 0.000) (Figure 8), indicating the underlying interactions between vascular geometry and hemodynamics.

In the univariate logistic model, larger post-PTAS vessel tortuosity (*P* = 0.012), larger post-PTAS vessel angulation (*P* = 0.053), lower post-PTAS PR (*P* = 0.025), and smaller Δ tortuosity (*P* = 0.018), as well as smaller Δ angulation (*P* = 0.027), were closely related with ISR and should be consequently taken into account in the multivariate logistic regression. However, because post-PTAS tortuosity and Δ tortuosity were intrinsically related, which also applied to post-PTAS angulation and Δ angulation, and there was a negative linear correlation between vessel tortuosity and PR after PTAS, we included only Δ tortuosity, Δ angulation, and post-PTAS PR in the multivariate logistic regression. It turned out that smaller Δ tortuosity (odds ratio, 0.00; 95% confidence interval, 0.00–0.02; *P* = 0.038) was an independent risk factor of ISR in our multivariate model, and post-PTAS translesional PR was also a predictive factor of marginal significance (odds ratio, 0.00; 95% confidence interval, 0.00–1.34; *P* = 0.059) (Table 6).

## 4. Discussion

The current study was among the first studies using CFD to investigate the roles of hemodynamics and vessel geometry in governing ISR risk in severe ICAS patients after PTAS. Establishing simplified CFD models with generic blood properties and individualized boundary conditions extracted from transcranial Doppler, this article found that local hemodynamic and geometric features of ICAS lesions were significantly influenced by PTAS and played an important role in the occurrence of ISR.

It had been previously shown that vessel morphology and local hemodynamics were closely related and played an important role in the initiation and development of various cerebrovascular diseases. In addition to systemic risk factors, atherosclerosis was a chronic and systemic inflammatory disease with the interactions of hemodynamic, geometrical, and biological factors [27, 28]. Stent implantation induced vessel straightening, significantly decreased vessel curvature, remodeled the vessel, and changed hemodynamic patterns [10, 29]. In coronary and carotid atherosclerosis, stenting showed its ability to change the vessel geometry and the local hemodynamics [23, 24, 30]. In intracranial arteries, previous studies have described the effect of stent-induced straightening of vessels [31] and vascular angel remodeling [32–34] during stent-assisted coiling of intracranial aneurysms. With five PTAS cases, Schirmer and Malek described the WSS dynamic fluctuations in ICAS using CFD, showing the complex dynamic directional and amplitude oscillations across the lesion, which could be normalized by stenting [9]. The geometric and hemodynamic changing ability of stents was also proved by the current study in ICAS patients. PTAS resulted in significant decrease of vessel tortuosity (0.09 vs. 0.01, *P* = 0.000) and vessel angulation (51.11° vs. 15.97°, *P* = 0.000), elevation of PR (0.07 vs. 0.62, *P* = 0.000) and reduction of WSSR (13.93 vs. 2.90, *P* = 0.000) through stenotic lesions. In stent coiling patients, with the passage of time, these stents showed persistent self-straightening tendency and continually exerted on the cerebral vasculature, leading to longer-term delayed angular and vascular remodeling [32]. In the current study of ICAS patients, during the follow-up period, the remodeling of vessel geometry persisted because of the continuous outwardly directed radial force of stents, but the geometrical parameters did not show much difference compared with immediate poststenting vessel angulation (*P* = 0.112) and tortuosity (*P* = 0.575). In PTAS, the balloon inflation also attributed a lot to the vascular remodeling, which was absent in stent coiling, indicating that the most striking geometry change might occur during the intervention process for ICAS patients instead of during the early follow-up for intracranial aneurysm patients [32].

In-stent restenosis could be caused by four key processes following stenting: thrombus formation, arterial inflammation, neointimal hyperplasia (NIH), and remodeling. NIH was the predominant attributor [21]. The balloon inflation and stent deployment inevitably resulted in endothelial disruption and the subsequent proliferation and activation of regional smooth muscle cells, thus causing NIH and ISR [35, 36]. The degree of NIH was linked directly to the severity of endothelial injury induced by the angioplasty balloon and intravascular stent. In coronary atherosclerotic lesions, quantitative angiographic analysis revealed a triphasic luminal response characterized by early restenosis (until 6 months), intermediate regression (6 months to 3 years), and late renarrowing (beyond 4 years), which could probably be explained by the fibrotic scar formation and reduction in matrix proteoglycans [37]. Similarly, in stenting for intracranial aneurysm treatment, dynamic and spontaneously resolvable ISR has also been reported [36, 38, 39]. However, regression of ISR has not been seen in ICAS yet, which was consistent with the current study. This divergence might be attributed to the difference in the incidence and natural history of ISR between stent-assisted coiling and PTAS [40].

Tortuosity of cerebral artery [26] and arteries in other body districts (e.g., coronary artery [41], carotid artery [42], and peripheral artery [43]) has been found to correlate with the development of atherosclerotic disease or thickening of wall intima. From the hemodynamic point of view, the increased tortuosity might induce disturbances of local hemodynamic environment characterized by low wall shear stress that have been demonstrated to associate with the initiation and progression of atherosclerosis [44–46]. For coronary [23, 47, 48] and carotid stents [11, 21, 24, 42, 49], geometry of the blood vessels, especially tortuosity, had been suggested to attribute to not only atherogenesis but also in-stent NIH [1]. The current study showed an ISR rate of 17.95% in severe ICAS patients and also revealed the important role of vessel tortuosity. The stented arteries with ISR were much more tortuous (0.06 vs. 0.05, *P* = 0.001), and the reduction of tortuosity caused by stenting (Δ tortuosity) was also much smaller (0.05 vs. 0.08, *P* = 0.006), which turned out to be the independent risk factor for ISR (*P* = 0.038).

Studies focusing on the hemodynamics of ICAS were still scarce because the cerebral artery had a smaller vascular caliber, a more complex and tortuous architecture of the arterial tree, and different histological features from coronary arteries. Translesional PR, calculated as the ratio of the pressures distal and proximal to an ICAS lesion obtained in a CFD model, had been proven to be highly correlated with invasive fractional flow ratio [50], a variable adapted from the coronary circulation and could be used to reflect the hemodynamic significance of ICAS, thus being a promising diagnostic parameter in cerebrovascular disorders [51]. It was an index that took into account of the degree of stenosis, lesion length, eccentricity, and other geometric features of a lesion, reflecting the fractional or residual flow across a stenotic artery, with lower values indicating hemodynamically more significant lesions [52, 53]. Translesional PR played an important role in sustaining cerebral perfusion in patients with symptomatic ICAS [54]. Lower PR at the ICAS lesion significantly increased the risk of recurrent stroke despite optimal medical treatment [55]. The current study also proved the important role of PR in ICAS lesions by revealing the borderline independent predictive value of lower PR for ISR after PTAS.

WSS was the tangential stress of the flowing blood on arterial wall, a major force on the endothelial surface. Physiological WSS modulated the endothelial functions, thus influencing the initiation and progression of atherosclerosis [56, 57]. And it was also related with ISR after coronary stenting [23, 47] and carotid stenting [24, 49]. For intracranial arteries, elevated focal WSS at ICAS lesions significantly increased the risk of recurrent stroke despite optimal medical treatment [55]. In the current study, both WSS and WSSR significantly decreased after PTAS but showed no relationship with ISR. However, there was a strong linear correlation between PG and WSS as well as PR and WSSR both before (*r*_s_ =0.750, *r*_s_ = −0.672) and after stenting (*r*_s_ =0.548, *r*_s_ = −0.566), which was also demonstrated by previous studies in ICAS [58] and coronary artery [30]. And because of the positive linear correlation between WSSR and vessel tortuosity after stenting, which was proven to be the independent predictor for ISR in ICAS, it was reasonable to deduce that WSS or WSSR could have some influence on ISR in ICAS, which might be proven by future studies with larger sample and more advanced CFD models.

The current study had several limitations. First, because of the retrospective nature, there was some bias that could be avoided, such as the patients' selection and the quantification of geometric and hemodynamic parameters. Second, the sample size was relatively small, which might lower the accuracy of the statistical analyses. Because of the controversial conclusions on the outcome of PTAS, the population of ICAS patients receiving PTAS was still not large, which could explain the small sample size of our study to some degree. Furthermore, only simplified CFD models with the diseased artery and adjacent arteries were reconstructed, and although individualized inlet velocity was adopted, uniform outlet conditions and blood properties were still used. Adopting patient-specific boundary conditions such as the proximal and distal pressure measured by the pressure wire and blood properties in CFD simulation might increase the accuracy of quantification of hemodynamic metrics. In order to offset the confounders, relative rather than absolute values in the current study were adopted for analysis. In future studies, more advanced CFD models might provide more information about the general and local hemodynamics of intracranial arteries. Moreover, morphological features or components of the plaques were not included in this study. Combination of CFD techniques and high-resolution magnetic resonance imaging was needed for further analysis.

## 5. Conclusion

The current study was among the first attempts to use CFD-based cerebral blood flow simulation methods to describe the geometric and hemodynamic changes caused by stent implantation, explore the possible relationships between vessel geometry and local hemodynamics in ICAS, and investigate the role of vessel geometry and hemodynamics played on ISR after PTAS. It turned out that stenting resulted in predominant change of vessel geometry and consequently influenced the local hemodynamics significantly. After PTAS, both translesional PR and WSSR were linearly correlated with vessel tortuosity, indicating interactions between vessel geometry and hemodynamics in ICAS. Δ Tortuosity turned out to be an independent risk factor for ISR, and ICAS lesions with lower translesional PR after PTAS demonstrated a somewhat higher rate of ISR, suggesting the predominant roles of vessel geometry and hemodynamics played in ISR. Further studies with larger sample size, more accurate CFD modeling and blood flow simulation, and multimodel neuroimaging evaluations would be needed.

## Figures and Tables

**Figure 1:** Research flow chart. ICAS: intracranial atherosclerotic stenosis; PTAS: percutaneous transluminal angioplasty and stenting; ISR: in-stent restenosis.

**Figure 2:** A patient-specific model reconstructed from DSA images and the generated centerlines of the proximal and distal vessel to the local stenosis before and after PTAS. The vessel angulation is referred to as the angle between the centerlines (displayed by dotted arrows). DSA: digital subtraction angiography; PTAS: percutaneous transluminal angioplasty and stenting.

**Figure 3:** Centerline extracted from the interested vessel. Vessel tortuosity is defined as *T*/*D* − 1, where *T*, equal to T1 + T2, is the length of the centerline between two points proximal and distal to the local stenosis, respectively, and *D* is the straight-line distance between these 2 points.

**Figure 4:** A patient-specific three-dimensional geometry of the arteries of interest reconstructed from DSA source images and the mesh created on the vessel surface and within the vessel lumen. DSA: digital subtraction angiography.

**Figure 5:** CFD models showing distribution of pressure, WSS, and SSR across a 90% stenotic lesion over the left MCA-M1 before and after PTAS. (a) Shows a significant decrease of pressure distal to the lesion and a significant elevated WSS and SSR adjacent to the stenotic throat before PTAS. (b) Displays increased pressure and decreased WSS and SSR adjacent to the stenotic throat after PTAS. CFD: computational fluid dynamics; WSS: wall shear stress; SSR: shear strain rate; MCA: middle cerebral artery; PTAS: percutaneous transluminal angioplasty and stenting.

**Figure 6:** (a, b) Show a 68-year-old man diagnosed with a severe right MCA-M1 stenosis, with pretreatment vessel angulation of 76.62°. After PTAS, the vessel angulation was 56.40°. 4 months later, vessel angulation was 51.53°. (c, d) Show a 62-year-old man having a severe basilar stenosis, with pretreatment vessel angulation of 35.65°. Following PTAS, vessel angulation changed to 19.76°. At 6.5-month follow-up, vessel angulation was 16.96°.

**Figure 7:** The scatterplots of correlations between hemodynamic indices. (a) Shows the correlation between WSS_stenotic-apex_ and PG before and after PTAS. (b) Shows the correlation between translesional PR and WSSR before and post PTAS. WSS: wall shear stress; PR: pressure ratio; WSSR: wall shear stress ratio; PTAS: percutaneous transluminal angioplasty and stenting.

**Figure 8:** The scatterplots of correlations between geometric and hemodynamic metrics. (a) Shows the correlation between vessel tortuosity and WSSR after PTAS. (b) Shows the correlation between vessel tortuosity and translational PR after PTAS. WSSR: wall shear stress ratio; PR: pressure ratio; PTAS: percutaneous transluminal angioplasty and stenting.

**Table 1:** Comparison of baseline characteristics between ICAS patients with ISR and no ISR.

Variables	Overall *n* = 39	No ISR *n* = 32	ISR *n* = 7	*P*
Age (y)	58.00 (50.00–65.00)	57.50 (50.50–64.50)	59.00 (49.00–65.00)	0.985
Male	22 (56.41)	16 (50.00)	6 (85.71)	0.113
Smoker	15 (38.41)	12 (37.50)	3 (42.86)	1.000
Hypertension	26 (66.67)	22 (68.75)	4 (57.14)	0.666
Diabetes mellitus	13 (33.33)	12 (37.50)	1 (14.29)	0.388
Coronary artery disease	4 (10.26)	4 (12.50)	0 (0.00)	1.000
Dyslipidemia	27 (69.23)	21 (65.63)	6 (85.71)	0.403
Glucose (mmol/L)	5.62 (5.02–6.67)	5.78 (5.09–6.84)	5.02 (5.00–5.63)	0.143
NIHSS at admission	0 (0–1)	0 (0–1)	0 (0–1)	0.578
Symptom				
Headache/dizziness	19 (48.72)	17 (53.13)	2 (28.57)	
Limb weakness	17 (43.59)	12 (37.50)	5 (71.43)	
Limb numbness	10 (25.64)	9 (28.13)	1 (14.29)	
Aphasia	10 (25.64)	8 (25.00)	2 (28.57)	
Ataxia	1 (2.56)	1 (3.13)	0 (0.00)	
Blurred vision	4 (10.26)	4 (12.50)	0 (0.00)	
ICAS lesion				0.413
ICA	2 (5.13)	1 (3.13)	1 (14.29)	
MCA	20 (51.28)	16 (50.00)	4 (57.14)	
BA	11 (28.21)	9 (28.13)	2 (28.57)	
VA	6 (15.38)	6 (18.75)	0 (0)	

BA: basilar artery; ICA: internal carotid artery; ICAS: intracranial atherosclerotic stenosis; ISR: in-stent restenosis; MCA: middle cerebral artery; NIHSS: National Institutes of Health Stroke Scale; VA: vertebral artery.

**Table 2:** Hemodynamic changes after PTAS.

Variables	Pre-PTAS	Post-PTAS	*P*
PR	0.07 (0.00 to 0.31)	0.62 (0.41 to 0.82)	*0.000*
Pressures_stenotic-apex_,(Pa)	−1.84∗10^4^ (−2.75∗10^5^ to −7.21∗10^3^)	1.47∗10^3^ (−3.14 to 4.19∗10^3^)	*0.000*
SSR_stenotic-apex_ (s^−1^)	9.84∗10^3^ (3.32∗10^3^ to 2.30∗10^4^)	2.49∗10^3^ (1.47∗10^3^ to 4.55∗10^3^)	*0.000*
WSS_stenotic-apex_ (Pa)	2.93∗10^2^ (1.61∗10^2^ to 8.74∗10^2^)	6.91∗10^1^ (3.51∗10^1^ to 1.11∗10^2^)	*0.000*
WSSR	13.93 (8.37 to 40.30)	2.90 (1.69 to 4.48)	*0.000*

PR: pressure ratio (PR = pressure_poststenotic_/pressure_prestenotic_); PTAS: percutaneous transluminal angioplasty and stenting; SSR: shear strain rate; WSS: wall shear stress; WSSR: wall shear strain ratio. (WSSR = WSS_stenotic−apex_/WSS_prestenotic_). Italic characters indicate *P* < 0.05.

**Table 3:** Vessel remodeling caused by PTAS.

	Tortuosity	Angulation (°)
Pre-PTAS	0.09 (0.06–0.13)	51.11 (40.07–67.27)
Post-PTAS	0.01 (0.00–0.03)	15.97 (0.00–36.16)
Follow-up	0.01 (0.00–0.03)	21.46 (0.00–31.34)
*P*_1_ value	*0.000*	*0.000*
*P*_2_ value	*0.000*	*0.000*
*P*_3_ value	0.112	0.575

PTAS: percutaneous transluminal angioplasty and stenting; *P*_1_: *P* value of comparison between pre-PTAS and post-PTAS; *P*_2_: *P* value of comparison between pre-PTAS and angiographic follow-up; *P*_3_: *P* value of comparison between post-PTAS and angiographic follow-up. Italic characters indicate *P* < 0.05.

**Table 4:** Comparison of geometric and hemodynamic parameters between ISR and no ISR lesions.

Variables	Overall *n* = 39	No ISR *n* = 32	ISR *n* = 7	*P*
Tortuosity				
Pre-PTAS	0.09 (0.06–0.13)	0.10 (0.06–0.13)	0.08 (0.07–0.15)	0.661
Post-PTAS	0.01 (0.00–0.03)	0.05 (0.00–0.01)	0.06 (0.02–0.10)	*0.001*
Δ tortuosity	0.08 (0.05–0.11)	0.08 (0.06–0.12)	0.05 (0.02–0.06)	*0.006*
Angulation (°)				
Pre-PTAS	51.11 (40.07–67.27)	53.00 (40.48–66.55)	47.11 (37.81–68.57)	0.826
Post-PTAS	15.97 (0.00–36.16)	13.01 (0.00–32.90)	36.16 (8.57–62.57)	0.096
Δ angulation (°)	31.76 (18.29–41.27)	33.53 (22.85–44.05)	14.08 (6.00–29.24)	*0.016*
PR				
Pre-PTAS	0.07 (0.00–0.31)	0.08 (0.01–0.27)	0.01 (0.00–0.58)	0.884
Post-PTAS	0.62 (0.41–0.82)	0.67 (0.50–0.89)	0.36 (0.05–0.62)	*0.024*
Pressure_stenotic-apex_ (Pa)				
Pre-PTAS	−1.84∗10^4^ (−2.75∗10^5^ to −7.21∗10^3^)	−3.71∗10^4^ (−3.95∗10^5^ to −7.75∗10^3^)	−1.27∗10^4^ (−4.27∗10^4^ to −5.19∗10^3^	0.487
Post-PTAS	1.47∗10^3^ (−3.14 to 4.19∗10^3^)	2.22∗10^3^ (1.72∗10^1^ to 4.66∗10^3^)	6.49∗10^2^ (−1.81∗10^2^ to 2.42∗10^3^)	0.442
WSS_stenotic-apex_ (Pa)				
Pre-PTAS	2.93∗10^2^ (1.61∗10^2^ to 8.74∗10^2^)	3.28∗10^2^ (1.57∗10^2^ to 9.16∗10^2^)	2.28∗10^2^ (2.08∗10^2^ to 3.06∗10^2^)	0.534
Post-PTAS	6.91∗10^1^ (3.51∗10^1^ to 1.11∗10^2^)	7.02∗10^1^ (3.32∗10^1^ to 1.11∗10^2^)	5.53∗10^1^ (4.31∗10^1^ to 1.97∗10^2^)	0.798
WSSR				
Pre-PTAS	13.93 (8.37 to 40.30)	13.70 (7.90 to 39.77)	19.97 (10.41 to 48.39)	0.634
Post-PTAS	2.90 (1.69 to 4.48)	2.64 (1.58 to 4.41)	3.60 (2.34 to 5.68)	0.188
SSR_stenotic-apex_, (s^−1^)				
Pre-PTAS	9.84∗10^3^ (3.32∗10^3^ to 2.30∗10^4^)	1.06∗10^4^ (2.97∗10^3^ to 2.32∗10^4^)	7.91∗10^3^ (4.77∗10^3^ to 1.17∗10^4^)	0.742
Post-PTAS	2.49∗10^3^ (1.47∗10^3^ to 4.55∗10^3^)	2.52∗10^3^ (1.55∗10^3^ to 4.05∗10^3^)	2.28∗10^3^ (1.30∗10^3^ to 8.11∗10^3^)	0.971

*Δ* angulation: pre − PTAS angulation − post − PTAS angulation; ISR: in-stent restenosis; PR: pressure ratio (PR = pressure_poststenotic_/pressure_prestenotic_); PTAS: percutaneous transluminal angioplasty and stenting; WSS: wall shear stress; WSSR: wall shear stress ratio (WSSR = WSS_stenotic−apex_/WSS_prestenotic_); Δ tortuosity: pre − PTAS tortuosity − post − PTAS tortuosity. Italic characters indicate *P* < 0.05.

**Table 5:** Linear correlation between indices of vessel geometry and hemodynamics of ICAS.

Variable 1	Variable 2	*P*	*r*
Pre-PTAS PR	Pre-PTAS WSSR	*0.000*	−0.672
Post-PTAS PR	Post-PTAS WSSR	*0.000*	−0.566
Post-PTAS tortuosity	Post-PTAS PR	*0.000*	−0.673
Post-PTAS tortuosity	Post-PTAS WSSR	*0.000*	0.547

ISR: in-stent restenosis; PR: pressure ratio (PR = pressure_poststenotic_/pressure_prestenotic_); PTAS: percutaneous transluminal angioplasty and stenting; WSS: wall shear stress; WSSR: wall shear stress ratio (WSSR = WSS_stenotic−apex_/WSS_prestenotic_). Italic characters indicate *P* < 0.05.

**Table 6:** Univariate and multivariate logistic regression analyses for associations between geometric and hemodynamic metrics of ICAS and ISR after PTAS.

Variables	No-ISR (*n* = 32)	ISR (*n* = 7)	Unadjusted	Adjusted	
			*P*	Odds ratio (95% confidence interval)	*P*
Male	16 (50.00)	6 (85.71)	0.115		
Age (y)	57.50 (50.50–64.50)	59.00 (49.00–65.00)	0.984		
Hypertension	22 (68.75)	4 (57.14)	0.557		
Diabetes mellitus	12 (37.50)	1 (14.29)	0.261		
Coronary artery disease	4 (12.50)	0 (0.00)	0.999		
Dyslipidemia	21 (65.63)	6 (85.71)	0.316		
Glucose (mmol/L)	5.78 (5.09–6.84)	5.02 (5.00–5.63)	0.186		
Smoker	12 (37.50)	3 (42.86)	0.792		
Post-PTAS tortuosity	0.05 (0.00–0.01)	0.06 (0.02–0.10)	*0.012*		
Δ tortuosity	0.08 (0.06–0.12)	0.05 (0.02–0.06)	*0.018*	0.00 (0.00–0.02)	**0.038**
Post-PTAS angulation (°)	13.01 (0.00–32.90)	36.16 (8.57–62.57)	*0.053*		
Δ angulation (°)	33.53 (22.85–44.05)	14.08 (6.00–29.24)	*0.027*	1.02 (0.89–1.16)	0.772
Post-PTAS PR	0.67 (0.50–0.89)	0.36 (0.05–0.62)	*0.025*	0.00 (0.00–1.34)	0.059
Post-PTAS pressure (Pa)	2.22∗10^3^ (1.72∗10^1^ to 4.66∗10^3^)	6.49∗10^2^ (−1.81∗10^2^ to 2.42∗10^3^)	0.756		
Post-PTAS SSR (s^−1^)	2.52∗10^3^ (1.55∗10^3^ to 4.05∗10^3^)	2.28∗10^3^ (1.30∗10^3^ to 8.11∗10^3^)	0.843		
Post-PTAS WSS (Pa)	7.02∗10^1^ (3.32∗10^1^ to 1.11∗10^2^)	5.53∗10^1^ (4.31∗10^1^ to 1.97∗10^2^)	0.720		
Post-PTAS WSSR	2.64 (1.58 to 4.41)	3.60 (2.34 to 5.68)	0.441		

Δ angulation: pre − PTAS angulation − post − PTAS angulation; ISR: in-stent restenosis; PR: pressure ratio (PR = pressure_poststenotic_/pressure_prestenotic_); PTAS: percutaneous transluminal angioplasty and stenting; WSS: wall shear stress; WSSR: wall shear stress ratio (WSSR = WSS_stenotic−apex_/WSS_prestenotic_); Δtortuosity = pre − PTAS tortuosity − post − PTAS tortuosity. Italic characters indicate unadjusted *P* < 0.1. Bold characters indicate adjusted *P* < 0.05.

## Data Availability

The datasets generated during the current study are available from the corresponding author on reasonable request.

## Supplementary Materials

Supplementary Materials Supplemental material: STROBE Statement—checklist of items that should be included in reports of observational studies.
